This article has been retracted.

# Analgesic Effects of Different *κ*-Receptor Agonists Used in Daytime Laparoscopic Cholecystectomy

**DOI:** 10.1155/2021/2396008

**Published:** 2021-12-29

**Authors:** Wanjun Zhou, Jiawu Wang, Chengyun Hu, Feibiao Dai, Zhetao Zhang, Chuanyao Li, Chaoliang Tang, Yanhu Xie

**Affiliations:** ^1^Department of Anesthesiology, The First Affiliated Hospital of USTC, Division of Life Sciences and Medicine, University of Science and Technology of China, Hefei, Anhui 230001, China; ^2^Department of Pharmacy, The First Affiliated Hospital of USTC, Division of Life Sciences and Medicine, University of Science and Technology of China, Hefei, Anhui 230036, China

## Abstract

**Background:**

Comparing the effect of two different *κ*-receptor agonists, nalbuphine and oxycodone, and regular morphine in patients for prophylactic analgesia of acute pain after daytime laparoscopic cholecystectomy.

**Methods:**

One hundred and twenty-four patients undergoing laparoscopic cholecystectomy were randomly allocated to receive nalbuphine (group N), oxycodone (group O), and morphine (group M). The three groups were all given intravenous injection (iv.) of 0.15 mg/kg injection before incision and 0.05 mg/kg injection at the end of pneumoperitoneum. The Visual Analogue Scale (VAS) scores (incision, visceral, and shoulder) and Ramsay sedation scores at 1, 2, 4, 8, 12, 16, 20, and 24 hours after surgery, the time of extubation, the incidence of postoperative adverse events, the satisfaction of pain treatment, and the duration of stay after surgery were all recorded.

**Results:**

Compared with group M, the VAS scores of visceral pain at rest decreased in group N and group O at 1-8 h after surgery (*P* < 0.05). The VAS scores of visceral pain at movement in group N decreased longer than those in group O (*P* < 0.05). Compared with that of group M, the postoperative time in Ramsay sedation score of group O increased longer than that of group N (*P* < 0.05). Compared with group N, patients had worse sleep quality in group O, longer length of stay in group M, and lower satisfaction in both groups.

**Conclusion:**

Compared with morphine, prophylactic use of the *κ*-receptor agonists, nalbuphine and oxycodone, during laparoscopic cholecystectomy can reduce postoperative visceral pain. Furthermore, the nalbuphine group had fewer adverse reactions, better analgesia, and better satisfaction.

## 1. Introduction

In recent years, with the rapid development of enhanced recovery after surgery (ERAS), day surgery has emerged. Among them, enhanced recovery and adequate analgesia are an essential part of increasing the rate of day surgery [1]. Laparoscopic cholecystectomy (LC) is a typical example of laparoscopic surgery. However, about 80% of patients undergoing LC experience moderate to severe postoperative acute pain due to pneumoperitoneum and intraoperative trauma [2]. Under the influence of this pain, it may cause prolonged wound healing and infection. Postoperative cognitive impairment, prolonging the length of stay, or even developing chronic pain may also appear; these are the main reasons why LC cannot be included in the day surgery [3].

A variety of methods can be used for postoperative analgesia of LC, of which local anesthetic incision infiltration was used for somatic pain, besides warming and humidifying the carbon dioxide (CO_2_) used for referred pain [4, 5]. For patients, suffering from visceral pain for day LC, weaker opioids are recommended currently [6]. As a classical *μ*-opioid receptor, morphine is a very effective measure of opioid pharmacodynamics, with a definite analgesic effect. However, it has a short duration of action and causes numerous adverse effects, which may not be suitable for ambulatory surgery [7]. Nalbuphine and oxycodone are two new opioid analgesics. Both, activated *κ*-opioid receptor, have been a hot topic of research in recent years for the treatment of perioperative visceral pain. Opioids act by binding to receptors in the central nervous system, peripheral nervous system, and many other organ systems. Through studies, peripheral *κ*-opioid receptors were found to be widely distributed in the viscera, which may be the main reason for the superiority of *κ*-opioids in the treatment of visceral pain [8]. The *κ*-opioid receptor has a high concentration in the spinal cord and its agonist, nalbuphine with oxycodone, inducing only mild respiratory depression with a ceiling effect. In addition, *κ* receptors with analgesic and sedative effects are not cross-tolerant with *μ* receptors, and the analgesic effect is superimposed [9]. Oxycodone is a semisynthetic opioid analgesic and a *κ*_2_ receptor agonist with low affinity for *μ* receptors, which is widely used in clinic [10]. As a *κ*-receptor agonist-antagonist, nalbuphine agonizes *κ* receptors to achieve analgesia, while antagonizing *μ* receptors to reduce opioid side effects, and is good postoperative analgesia and a good antagonist of opioid-induced adverse reactions [9].

However, the analgesic effects of nalbuphine and oxycodone are comparable to morphine by the results of current clinical practice. Still, the safety of both is better than morphine in terms of specific side effects [11, 12]. There are no definitive clinical studies suggesting which of these two *κ*-receptor agonists is more effective for prophylactic analgesia for acute postoperative pain after LC. This is a prospective randomized controlled study, which is aimed at comparing the analgesic effects and occurrence of adverse effects of nalbuphine and oxycodone for prophylactic analgesia in LC. Then, select a more suitable drug to provide a reference for future clinical practice in the day surgery mode of LC.

## 2. Methods

### 2.1. Demographic Parameters

One hundred and twenty-four patients, who underwent LC in the First Affiliated Hospital of University of Science and Technology of China, were selected from May 2019 to June 2020. Patients aged 18-65 yr, with a body mass index (BMI) of 18.5-30 kg/m^2^, scheduled for daytime LC, and with American Society of Anesthesiologists (ASA) physical status of I or II, were eligible. Patients were excluded if they had severe respiratory and circulatory diseases, nervous system diseases, mental and psychological diseases, obvious abnormal liver and kidney functions, opioid allergy, or long-term abuse of drugs (including antineoplastic and analgesics) or if they had intraoperative conversion to open surgery. The study was approved by the Ethics Committee of the First Affiliated Hospital of USTC (serial number, 2019-Q (H)-001), and written informed consent was obtained from all subjects or the legal surrogate.

### 2.2. Experimental Grouping

Patients were randomly divided into three groups (nalbuphine group, oxycodone group, and morphine group) at an allocation ratio of 1 : 1 : 1 via block randomization generated by computer-generated randomization software. Group allocations were sealed in sequentially numbered, opaque envelopes that were opened by one trained study personnel after the induction of general anesthesia. Each envelope contained the group allocation with instructions of analgesic for the attending anesthesiologists.

The nalbuphine group (group N) was given 0.15 mg/kg nalbuphine injection before skin cutting and 0.05 mg/kg nalbuphine injection after surgery. The oxycodone group (group O) was given 0.15 mg/kg oxycodone injection before skin cutting and 0.05 mg/kg oxycodone injection after surgery. The morphine group (group M) was given 0.15 mg/kg morphine injection before skin cutting and 0.05 mg/kg morphine injection after surgery.

### 2.3. Anesthesia

General anesthesia was induced with by 1 *μ*g/kg remifentanil and 0.2-0.4 mg/kg etomidate. Tracheal intubation was facilitated by 0.6 mg/kg rocuronium. Then, an I-gel laryngeal mask was placed, and a gastric tube was placed after 90 s. Mechanical ventilation was performed with a tidal volume of 6-8 ml/kg, respiratory rate of 10-14 times/min, inhalation/respiration ratio of 1/2, inhalation oxygen concentration of 50%, and End-tidal carbon dioxide partial pressure (P_ET_CO_2_) maintained between 35 and 45 mmHg. Experimental analgesic (diluted to 10 ml, iv.) was given before skin cutting. Anesthesia was maintained in target controlled infusion with propofol (2.0-4.0 *μ*g/ml) and remifentanil (2.0-4.0 ng/ml), and plasma concentrations of propofol and remifentanil were adjusted to maintain a level of 27-56 (stage E0-D1) and according to 20% variations in blood pressure and/or heart rate compared with basal values. Rocuronium was given at 10 mg per injection as needed. After the operation, all anesthesia drugs were stopped and experimental analgesics were given (diluted to 10 ml, iv.). When the skin was sutured, 10 ml ropivacaine (0.5%) was given through the skin incision to infiltrate the local anesthesia layer by layer.

### 2.4. Surgery

All groups of patients were operated by the same group of surgeons, using the 3-hole method, and the pneumoperitoneum pressure was 14 mmHg (warming and humidifying the CO_2_). An abdominal drainage tube should not be placed after surgery unless in special circumstances. After surgery, the residual CO_2_ was deflated carefully.

### 2.5. Rescue Analgesics

In cases where patients experienced significant postoperative pain (VAS ≥ 4), rescue analgesics (50 mg flurbiprofen axetil injection per time) were recommended for patients. The use of rescue analgesics was recorded.

### 2.6. Observation Target

The patients' demographic parameters, anesthesia time, and extubation time were recorded. Before surgery, the patients were instructed to use a 100 mm VAS [0-10, 0 = no pain and 10 = worst pain imaginable] to rate the following three pain components: incisional pain was defined as a superficial pain, wound pain, or pain located in the abdominal wall. Visceral pain was defined as pain inside the abdomen. Shoulder pain was defined as a sensation of pain in the shoulder. Follow-up evaluations were conducted at 1, 2, 4, 8, 12, 16, 20, and 24 h postoperatively by anesthesiologists blinded to grouping. The degree of incision pain and visceral pain was evaluated when resting and in motion (cough and deep breathing), respectively. And record the Ramsay sedation score (1—patient is anxious and agitated or restless or both; 2—patient is cooperative, orientated, and tranquil; 3—patient responds to commands only; asleep levels were dependent on the patient's response to a light glabellar tap or loud auditory stimulus; 4—there is a brisk response; 5—there is a sluggish response; and 6—there is no response vital signs and sleep) [13]. The pain treatment satisfaction scale (PTSS) (PTSS, 0 = no satisfaction to 10 = complete satisfaction) [14] and major adverse effects such as postoperative nausea and vomiting (PONV) (PONV four-point scale: 1 = no nausea; 2 = mild nausea; 3 = severe nausea requiring antiemetic; and 4 = retching and/or vomiting) [15] and minor adverse effects such as hypoxemia, drowsiness, dizziness, skin pruritus, and urinary retention were recorded. Rescue analgesia within 24 h after surgery and unplanned discharge (the length of stay ≥ 24 h after surgery) was also used.

### 2.7. Sample Size

The power calculation for the study was based on the VAS of visceral pain at rest at 1 h after surgery, which was our primary outcome. A pilot study involving 8 patients at our center found that the mean ± standard deviation (SD) of the VAS of visceral pain at rest at 1 h after surgery was 4.5 ± 1.8. In a sample size of 40 patients, a clinically significant reduction of 30% in the VAS of visceral pain at rest at 1 h after surgery at a power of 95% was observed, with a two-sided significance level of 0.05. To compensate for the possibility of dropouts, we recruited a total of 132 patients, with 44 patients per group.

### 2.8. Statistical Analysis

The SPSS 22.6 software was used for statistical analyses. Distribution of variables was assessed using the Kolmogorov-Smirnov test, while homogeneity of variance was evaluated using Levene's test. Quantitative data were expressed as the $\text{mean}\pm \text{standard deviations }\left(\bar{x}\pm \text{s}\right)$ or medians and interquartile ranges. The enumeration data are represented by the number of examples. If the measurement data conform to the normal distribution, the analysis of variance (ANOVA) for repeated measurements is adopted, while Bonferroni's method was used to compare groups. If they do not conform, the one-way ANOVA of Kruskal Wallis test is adopted and Bonferroni's method was used to compare groups. The enumeration data were performed by *χ*^2^ test. *P* < 0.05 was considered to be statistically significant.

## 3. Results

### 3.1. Quantitative Analysis of Patients

One hundred and thirty-two patients were recruited from May 2019 to June 2020. Three patients in group M dropped out of the study, one converted to open surgery, and two did not complete date collection. Two patients in group N dropped out of the study, due to failure to complete data collection. Three patients in group O dropped out of the study, two converted to open surgery, and one did not complete date collection. One hundred and twenty-four patients completed the study: 41 in group M, 42 in group N, and 41 in group O (Figure 1). There was no statistically significant difference in the demographic parameters among the 3 groups (*P* > 0.05), and there was comparability between the three groups. (Table 1).

### 3.2. Hemodynamic Variables

There were no statistically significant differences in heart rate, mean arterial pressure, and oxygen saturation among the three groups at each time point (Table 2).

### 3.3. The VAS Score (at Rest and Movement)

There was no significant difference in the VAS score of incision pain (at rest and movement) among the three groups. Compared with group M, the VAS score of visceral pain at rest in group N and group O decreased 1-8 h after surgery (*P* < 0.05). The VAS score of visceral pain at movement in group N was significantly decreased 2-20 h after surgery, and that in group O was significantly decreased 2-8 h after surgery (*P* < 0.05). There was no statistical significance in VAS scores of shoulder pain among the three groups (Figure 2, Table 3).

### 3.4. Anesthesia Recovery

There was no significant difference in extubation time among the three groups. Compared with group N, patients had worse sleep quality in group O and lower pain treatment satisfaction in other two groups (*P* < 0.05), while the differences between groups M and O were not statistically significant. In the case of using rescue analgesia within 24 h postoperatively, that in groups N, O, and M increased sequentially; however, the differences were not statistically significant. Unplanned discharges of patients were significantly reduced in the group N compared to group M. (Table 4). Compared with group M, Ramsay sedation score of group O was significantly increased 1-8 h after surgery, while that of group N was significantly increased 1-4 h after surgery (*P* < 0.05) (Figure 3).

### 3.5. Postoperative Adverse Events

The occurrence of PONV in patients was significantly reduced in group N compared to group M (*P* < 0.05), and the difference was not statistically significant in group O compared to both group M and group N. The occurrence of other side effects was reduced in both group O and group N, in which 7 patients in group M had significantly more pruritus than the other two groups, and 18 patients in group M had significantly more dizziness than 4 patients in group N. The differences were all statistically significant (*P* < 0.05) (Table 5).

## 4. Discussion

This study mainly found that compared with morphine, preventive use of *κ*-receptor agonists, nalbuphine and oxycodone, in LC can significantly reduce postoperative visceral pain. The nalbuphine group has fewer complications such as postoperative dizziness, nausea, and vomiting and has better effect in reducing early postoperative pain and better patient satisfaction.

LC has the advantages of minimally invasive and quick recovery. With the deepening of ERAS concept, daytime surgery, which completes admission, discharge and corresponding surgery, and operation within one working day, arises at the historic moment. Nowadays, more and more clinicians use LC in daytime surgery. The development of daytime surgery would speed up patient turnover, reduce waiting time, reduce the risk of nosocomial infection, improve the use efficiency of medical resources, and reduce various expenses. A standardized daytime surgery system has clinical and economic win-win benefits [1]. However, postoperative pain is the main factor leading to delayed discharge of daytime surgery patients [16]. Previous studies have shown that postoperative pain mainly consists of three components: abdominal incision pain related to the incisional trauma at the port sites, visceral pain associated with tissue injury due to gallbladder dissection, and the stretching of nerve endings in the peritoneal cavity, and right shoulder pain is referred by diaphragmatic stretching. Among these pains, visceral pain is worse than incision and shoulder pain in postoperative acute pain [17]. Nalbuphine and oxycodone are the research hotspots in the treatment of postoperative visceral pain in recent years because of their agonistic effects on *κ*-opioid receptors.

This study found that there was no significant difference in VAS scores of incision pain (at rest and movement) among the three groups of patients, which may be related to the layer-by-layer infiltration of 0.5% ropivacaine in the three groups of patients. It also indicates that the two *κ*-receptor agonists may have the same analgesic effect on abdominal incision pain as morphine. The VAS scores of visceral pain (at rest and movement) in oxycodone and nalbuphine groups were significantly reduced within 2-8 hours after operation. It is suggested that the analgesic effect of oxycodone and nalbuphine on visceral pain may be better than that of morphine. This is because the two *κ*-receptor agonists inhibit the sensitization of peripheral pain *κ*-opioid receptors and the excitatory neurotransmission between the afferent nerves expressing *κ*-opioid receptors and the superficial neurons of the spinal cord that process pain signals. These functional *κ*-opioid receptors have abundant innervation not only for skin but also for visceral organs, which indicates that *κ*-opioid receptors are of great significance in inhibiting visceral pain [18].

On Ramsay sedation score, the mean value of morphine group was less than 2 at 1-16 hours after operation. It may be related to the imperfect analgesia in this group, which improves the arousal level and offsets the sedation induced by morphine. In an experimental pain study on sedation, it was also found that morphine had no effect on sedation variables in electroencephalograph [19]. Compared with the morphine group, the oxycodone group increased significantly 1-8 h after operation, while the nalbuphine group increased significantly 1-4 h after operation, both of which were more than 2 scores, which may be related to the sedative effect of both through central nervous system *κ*-opioid receptors [20].

The study also found some differences between the two *κ*-receptor agonists in terms of analgesic effect. Compared with that in the oxycodone group, VAS score of visceral pain at movement in the nalbuphine group was still significantly lower 12-20 h after operation. The reason may be that oxycodone is a semisynthetic opioid receptor agonist, which has double agonism of both *μ*-opioid receptors and *κ*-opioid receptors, and the half-life of oxycodone intravenous injection is 3.5 h. Nalbuphine, on the other hand, is a morphinan semisynthetic agonist-antagonist analgesic, which exerts pharmacological effects through agonist *κ*-opioid receptors and antagonist *μ*-opioid receptors with a half-life of 5 h. Although nalbuphine is an agonist antagonist, its analgesic effect is not weakened by *μ*-opioid receptors antagonism. This may be one of the reasons for the longer analgesic effect of nalbuphine [9, 20]. The expression and distribution of *κ*-opioid receptors are quite different among different internal organs, and their analgesic effect is mainly mediated by stimulating peripheral *κ*-opioid receptors. Under the condition of inflammation and pain sensitization, the peripheral analgesic effect of *κ*-opioid receptor agonists would be further enhanced. Oxycodone is a *κ*_2_-opioid receptor agonist with relatively low affinity to *μ*-opioid receptors, of which the *μ*-opioid receptor agonism is not strong. Nalbuphine mainly exerts analgesic effect through agonist *κ*-opioid receptors [10, 20]. Therefore, we speculate that the longer analgesic effect of nalbuphine may also be related to the stronger selectivity of nalbuphine to *κ*-opioid receptors. In addition, nalbuphine can also increase the density and activity of opioid *κ*-opioid receptors, and then improve the analgesic effect [21]. The specific mechanisms of these two scores need a further study. We give opioids in advance before skin incision to directly prevent noxious stimulation impulses from entering the center or directly inhibit the excitability of the central nervous system, reduce, or eliminate the sensitization of the central nervous system caused by adverse stimulation. It plays a preventive analgesic role and further prolongs the time limit of the two drugs.

In the past clinical practice, the dose limitation of opioids is precisely due to its agonism of *μ*-opioid receptors, which leads to respiratory depression, addiction, itching, nausea, and vomiting. This study also found that the incidence of postoperative adverse reactions in the morphine group was generally higher than that in the other two groups. Previous studies have inconsistent results in comparing the side effects of morphine and oxycodone. Yanagidate and Dohi found that morphine may have a higher incidence of nausea, vomiting, and skin pruritus [22]. However, other studies show that the side effects of the two drugs may not be significantly different [23, 24]. Pedersen et al. pointed out that morphine has lower incidence of adverse reactions and higher safety than oxycodone [25]. The total number of complications and the incidence of skin pruritus in the oxycodone group were significantly lower than those in the morphine group. Although the incidence of other adverse reactions (such as urinary retention, nausea and vomiting, respiratory depression, and dizziness) decreased, the difference was not statistically significant. However, the adverse reactions (skin pruritus, nausea and vomiting, and dizziness) in the nalbuphine group are significantly decreased than those in the morphine group. It is also consistent with the fact that nalbuphine has lower incidence of adverse reactions and higher safety than morphine mentioned in previous studies [9, 11]. This is because nalbuphine antagonist *μ*-opioid receptors can prevent or alleviate side effects such as skin pruritus, dizziness, nausea, and vomiting [26], while oxycodone with double *μ*-opioid receptors and *κ*-opioid receptors agonism may increase the occurrence of postoperative adverse reactions. Therefore, the nalbuphine group may be more advantageous in the prevention of adverse reactions than the other two groups.

Pain management is an important measure in Enhanced Recovery After Surgery (ERAS). There is a significant correlation between the number and severity of postoperative adverse reactions and the decline of patient-oriented results (such as recovery quality and patient satisfaction) [27]. Previous studies had also shown that the increase of postoperative pain and nausea is significantly related to the decline of immediate postoperative recovery quality [28]. The patient's daily life, rest, wound healing, and length of stay will be affected by severe PONV. As mentioned earlier, nalbuphine has the best analgesic effect among the three groups, and the incidence of adverse reactions such as dizziness, nausea, and vomiting and skin pruritus is reduced. This is consistent with the fact that the nalbuphine group has higher sleep quality, higher pain treatment satisfaction, and shorter length of stay than the other two groups. It indicates that preventive use of nalbuphine for LC patients has higher comfort than the other analgesics, which is more in line with ERAS concept, and may be a better analgesic choice for daytime development of laparoscopic surgery.

Postoperative release of inflammatory cytokines may lead to excessive stress, immunosuppression, pain sensitization, etc., which would aggravate postoperative pain and delay postoperative rehabilitation. This study did not measure cytokines by blood sampling and compared the effects of the different *κ*-receptor agonists on inhibiting the release of inflammatory cytokines after operation. These will be further explored in subsequent studies.

In conclusion, compared with morphine, postoperative visceral pain will be reduced significantly in prophylactic use of *κ*-receptor agonists, nalbuphine, and oxycodone in daytime LC. The nalbuphine group has fewer adverse reactions such as dizziness, nausea, and vomiting and has better effect in relieving early postoperative pain, which can improve patients' satisfaction with anesthesia and shorten length of stay. Therefore, it is more recommended to apply to daytime LC surgery.

## Figures and Tables

**Figure 1:** Flow diagram of patient recruitment.

**Figure 2:** Postoperative VAS pain score of incision pain (a) at rest and (b) at movement; VAS pain score of visceral pain (c) at rest and (d) at movement during a 24 h postoperative period. Data are the mean with standard deviation. ^∗^*P* < 0.05, group O compared with group M; ^#^*P* < 0.05, group N compared with group M.

**Figure 3:** Postoperative Ramsay sedation score during a 24 h postoperative period. Data are the mean with standard deviation. ^∗^*P* < 0.05, group O compared with group M; ^#^*P* < 0.05, group N compared with group M.

**Table 1:** The demographic parameters among the three groups.

Group	Patients (n)	Men/women (*n*)	Age (years)	BMI (kg/m^2^)	ASA I/II (*n*)	Time of operation (min)
M	41	13/28	45.1 ± 13.3	23.3 ± 2.4	29/12	56.3 ± 22.5
N	42	16/26	45.6 ± 10.0	23.8 ± 2.7	28/14	56.8 ± 24.3
O	41	15/26	47.3 ± 12.0	24.7 ± 2.6	28/13	56.2 ± 20.9

Values are given as the mean ± standard deviation or number of patients.

**Table 2:** Comparison of vital signs at different time points in three groups.

Group	Preoperative	Postoperative							
		1 h	2 h	4 h	8 h	12 h	16 h	20 h	24 h
Heart rate (times/min)									
M	77.0 ± 6.8	76.9 ± 8.1	77.8 ± 7.2	76.5 ± 5.4	75.6 ± 5.8	74.8 ± 6.2	74.2 ± 5.7	75.0 ± 6.3	75.2 ± 8.2
N	77.0 ± 8.6	76.5 ± 7.6	76.8 ± 8.5	75.0 ± 7.1	75.7 ± 7.2	74.2 ± 5.1	74.6 ± 7.9	74.6 ± 5.8	75.0 ± 6.9
O	75.5 ± 11.4	76.3 ± 9.8	76.0 ± 9.3	75.3 ± 8.2	74.9 ± 9.3	73.9 ± 8.0	74.8 ± 6.3	74.6 ± 7.0	75.5 ± 9.1
Mean arterial pressure (mmHg)									
M	92.0 ± 7.2	87.9 ± 8.6	87.7 ± 9.1	88.9 ± 6.9	88.5 ± 7.2	89.8 ± 8.8	88.3 ± 5.2	88.5 ± 7.3	90.8 ± 8.6
N	92.5 ± 8.3	85.2 ± 8.6	86.8 ± 7.7	86.2 ± 7.5	87.5 ± 6.8	88.2 ± 7.8	89.8 ± 9.2	90.5 ± 7.8	91.2 ± 6.8
O	92.3 ± 10.4	86.2 ± 8.8	86.0 ± 9.5	86.8 ± 7.2	88.9 ± 9.2	88.9 ± 8.6	89.6 ± 6.9	90.1 ± 8.0	90.5 ± 8.2
Oxygen saturation (%)									
M	97.3 ± 0.7	98.0 ± 0.8	98.9 ± 0.8	98.1 ± 1.0	97.1 ± 0.8	97.1 ± 0.8	97.1 ± 0.6	96.9 ± 0.8	97.2 ± 0.6
N	97.4 ± 0.8	98.9 ± 0.9	99.0 ± 0.9	98.8 ± 0.8	97.3 ± 0.6	97.3 ± 0.6	97.5 ± 0.8	97.3 ± 0.5	97.2 ± 0.7
O	96.9 ± 1.2	98.5 ± 1.4	98.5 ± 1.3	98.7 ± 0.9	96.7 ± 0.9	96.7 ± 0.9	97.2 ± 0.7	97.1 ± 0.7	96.8 ± 0.9

Values are given as the mean ± standard deviation.

**Table 3:** VAS scores in the shoulder among the three groups at different time points.

Group	Postoperative							
	1 h	2 h	4 h	8 h	12 h	16 h	20 h	24 h
M	0.0 ± 0.0	0.0 ± 0.0	0.0 ± 0.2	0.1 ± 0.3	0.0 ± 0.2	0.0 ± 0.0	0.0 ± 0.0	0.0 ± 0.0
N	0.0 ± 0.0	0.0 ± 0.0	0.1 ± 0.3	0.1 ± 0.4	0.1 ± 0.3	0.0 ± 0.2	0.0 ± 0.0	0.0 ± 0.0
O	0.0 ± 0.0	0.0 ± 0.0	0.0 ± 0.2	0.1 ± 0.3	0.1 ± 0.2	0.0 ± 0.0	0.0 ± 0.0	0.0 ± 0.0

Values are given as the mean ± standard deviation.

**Table 4:** The situation of extubation.

Group	Extubation time (min)	Sleep	Rescue analgesia [*n* (%)]	PTSS	Unplanned discharge [*n* (%)]
M	15.0 (7.0, 20.0)	2 (1, 2)	5 (12.2%)	7 (6, 8)^#^	15 (36.6%)^#^
N	11.0 (5.0, 21.3)	1 (1, 2)	1 (2.3%)	8 (7, 10)^∗^	3 (7.2%)^∗^
O	14.5 (7.8, 20.5)	2 (1, 2)^#^	3 (7.3%)	7 (4, 10)^#^	8 (19.5%)

Values are given as medians and interquartile ranges or number of patients (%). ^∗^*P* < 0.05 compared with group M; ^#^*P* < 0.05 compared with group N. Statistical criteria: sleep (1—good, 2—average, 3—poor, and 4—insomnia).

**Table 5:** The incidence of postoperative adverse reactions in the three groups.

Group	PONV scores	Pruritus (*n*)	Uroschesis (*n*)	Respiratory depression (*n*)	Dizziness (*n*)
M	2 (1, 2)^#^	7 (17%)	2 (5%)	1 (2%)	18 (44%)^#^
N	1 (1, 1)^∗^	0^∗^	0	0	4 (10%)^∗^
O	1 (1, 2)	1 (2%)^∗^	1 (2%)	0	9 (33%)

Values are given as medians and interquartile ranges or number of patients (%). ^∗^*P* < 0.05 compared with group M; ^#^*P* < 0.05 compared with group N.

## Data Availability

The data used to support the findings of this study are available from the corresponding author upon request.
